The article "Lactobacillus rhamnosus GG Colonization in Early Life Ameliorates Inflammaging of Offspring by Activating SIRT1/AMPK/PGC-1α Pathway" was published in 2021. Journal: Oxid Med Cell Longev.

# *Lactobacillus rhamnosus GG* Colonization in Early Life Ameliorates Inflammaging of Offspring by Activating SIRT1/AMPK/PGC-1*α* Pathway

**DOI:** 10.1155/2021/3328505

**Published:** 2021-11-11

**Authors:** Tianyu Liu, Xueli Song, Yaping An, Xuemei Wu, Wanru Zhang, Jia Li, Yue Sun, Ge Jin, Xiang Liu, Zixuan Guo, Bangmao Wang, Ping Lei, Hailong Cao

**Affiliations:** ^1^Department of Gastroenterology and Hepatology, Tianjin Medical University General Hospital, Tianjin Institute of Digestive Diseases, Tianjin Key Laboratory of Digestive Diseases, Tianjin, China; ^2^Department of Geriatrics, Tianjin Medical University General Hospital, Tianjin, China

## Abstract

Inflammaging refers to chronic, low-grade inflammation during aging, which contributes to the pathogenesis of age-related diseases. Studies have shown that probiotic intervention in the aging stage could delay aging-related disorders. However, whether the application of probiotics in early life could have antiaging effects on offspring was unknown. Here, we investigated the effects of *Lactobacillus rhamnosus GG* (*LGG*) colonization in early life on inflammaging of offspring. Pregnant mice with the same conception time were given *LGG* live bacteria (LC group) or *LGG* fixed bacteria (NC group) from the 18th day after pregnancy until natural birth. The progeny mice were treated with 10^7^ cfu of live or fixed LGG for 0-5 days after birth, respectively. *LGG* colonization could be detected in the feces of 3-week offspring. The 16S rRNA sequencing analysis of 3-week-old offspring showed that colonization of *LGG* in early life could alter the composition and diversity of gut microbiota. Interestingly, the beneficial effects of *LGG* colonization in early life on the microbiota lasted to 8 months old. The abundance of longevity-related bacteria (*Lactobacillus*, *Bifidobacterium*, and *Akkermansia muciniphila*) increased significantly in the *LGG* colonization group. In addition, *LGG* colonization increased the abundance of short-chain fatty acid- (SCFA-) producing bacteria and the production of cecal SCFAs. *LGG* colonization in early life protected the intestinal barrier, enhanced antioxidant defense, attenuated epithelial cell DNA damage, and inhibited intestinal low-grade inflammation in 8-month-old progeny mice. Mechanically, *LGG* could upregulate Sirtuin1 (SIRT1)/Adenosine 5′-monophosphate-activated protein kinase (AMPK)/Peroxisome proliferator-activated receptor *γ* coactivator 1-*α* (PGC-1*α*) pathway and repress activation of nuclear factor-kappa B (NF-*κ*B), while the protective effect of *LGG* was blunted after SIRT1 gene silencing. Together, *LGG* colonization in early life could ameliorate inflammaging of offspring, which would provide a new strategy for the prevention of age-related diseases.

## 1. Introduction

Aging is a complex process characterized by a continuous and progressive decline in physiological function and adaptive capacity, which increases the incidence of cancer and many chronic diseases [1, 2]. It is commonly believed that healthy aging and longevity are modulated by complex interactions between genetic and nongenetic (e.g., lifestyle, sociodemographics, and living situation) factors [3, 4], both of which are closely related to the gut microbiota.

In humans, about 100 trillion microbes inhabited in the nutrient-rich gut environment, the vast majority of which were nonpathogenic bacteria and maintained human health [5]. From birth, the adult-like gut microbiota community is established by the end of approximately the first 3 y of life and remains relatively stable throughout adult life [6]. This period is defined as the early stage of life, which is crucial to the health, metabolism, and ontogeny of an individual. The microbiota can be transmitted from mothers to infants through a variety of ways, including feces, vaginal delivery, skin, and breastfeeding. Therefore, maternal gut microbiota has a significant impact on the microbial composition of offspring [7]. However, the stability of gut microbiota may fluctuate with aging-related factors such as physiologic, lifestyle, and health status [8]. Compared with healthy adults, the microbiota diversity of the elderly is reduced, and the composition of the microbiota varies greatly among individuals [9]. These findings emphasize the crucial role of the microbial community in early life on regulating health status and lifespan.

Probiotics containing *Bifidobacterium* and *Lactobacillus* have shown beneficial effects on improving life expectancy and alleviating aging-related disorders by regulating gut microbiota composition and systemic immunity [10, 11]. Oral administration of *Lactobacillus plantarum HY7714* or *Bifidobacterium breve B-3* has been shown to be effective in preventing skin photoaging [12, 13]. Treatment with *Lactobacillus brevis OW38* in aged mice could ameliorate aging-associated colitis and memory disorders by inhibiting gut microbiota lipopolysaccharide (LPS) production, NF-*κ*B activation, and p16 expression [14]. Supplementation with *Lactobacillus plantarum WCFS1* prevented the age-related decline in the colon mucus barrier [15]. *LGG* is a gram-positive bacterium isolated from the healthy human intestinal tract and has strong adhesive properties to intestinal cells [16, 17]. *LGG* has been widely used as a nutritional supplement for pregnant women and infants. Clinical studies have shown that perinatal *LGG* administration to mothers was effective to prevent eczema in children at high risk [18, 19], and feeding formulas supplemented with *LGG* to term infants could preferably support their normal growth [20].

*LGG* promotes anti-inflammatory pathways of the resident microbes [21], but the preventive effects of *LGG* in early life on aging-related disorders have not been well elucidated. Our present study described how *LGG* colonization in neonatal mice improves the health status at the early phase of aging, suggesting that *LGG* colonization in early life may be a novel prevention strategy for age-related conditions.

## 2. Materials and Methods

### 2.1. Mice and LGG Treatment

Live *LGG* (ATCC53103, USA) was cultured in Lactobacillus MRS broth. Glutaraldehyde-fixed *LGG* was performed according to a previous study [17]. A total of 20 adult C57BL/6 female mice (8 weeks of age) were purchased from Beijing HFK Bioscience Co., Ltd., and housed 5 per cage under specific pathogen-free (SPF) environment. The animal rooms were supplied with 100% HEPA-filtered air at 15 air changes per hour, and the normal temperature was controlled between 20 and 26°C. Mice were fed with a standard rodent chow diet and maintained with a natural light-dark cycle (12 h light and 12 h dark). All mice consumed regular sterilized drinking water ad libitum, and the water was changed weekly or as required. After 2 weeks of acclimation, they were mated with C57BL/6 males, and all the 18 pregnant mice with the same conception time were randomly divided into two groups and gavaged with 10^8^ cfu live *LGG* or fixed *LGG* from the gestational day 18 until natural birth. Subsequently, all offspring gave birth by vaginal delivery and we got 18 pups in the NC group (8 males and 10 females) and 20 pups (9 males and 11 females) in the LC group. To avoid the differences due to sex, we chose 14 offspring (7 males and 7 females) randomly in each group for the study. From the first day after birth, the offspring mice were fed with 10^7^ cfu live *LGG* or fixed *LGG* for 5 consecutive days. Seven mice (3 males and 4 females) were randomly chosen and killed from each group in the third week, and the rest of remaining mice were sacrificed at the eighth month. All animal experiments have been evaluated and approved by the Animal Ethical and Welfare Committee of Tianjin Medical University.

### 2.2. LGG Colonization Detection

We collected the feces of 3-week-old offspring to detect the colonization of *LGG*. Feces were cultured in MRS broth, and genomic DNA of cultured bacteria was extracted using DNA Rapid Extraction Kit (Tiangen, China) and then was used for polymerase chain reaction (PCR) amplification of 16S rRNA gene using *LGG*-specific primers (Table 1). The migration profile of PCR-amplified products was determined by denaturing gradient gel electrophoresis (DGGE) method. The genomic DNA of *LGG* was used as control.

### 2.3. Intestinal Tissue Processing

For C57BL/6 mice, 6 to 12 months was defined as the early phase of aging [22]. Mice were sacrificed at the end of the 8-month feeding period, and cecal contents were collected. The small intestinal and colon tissues were isolated and rinsed with ice-cold phosphate-buffered saline (PBS) solution. Parts of the tissues were immediately stored at -80°C in a refrigerator for further RNA and protein extraction, and the rest was embedded into Swiss rolls in paraffin for further pathological evaluation. Fresh stool pellets were collected before being sacrificed for gut microbiota analysis.

### 2.4. Histopathology and Immunohistochemistry Analysis

The paraffin-embedded intestinal sections were deparaffinized. Hematoxylin-eosin (HE) staining was performed to evaluate intestinal development by measuring villus/crypt length. For immunohistochemistry (IHC) staining, deparaffinized sections were incubated with the following primary antibodies overnight at 4°C: MUC2 (Santa Cruz Biotechnology, Inc.), GPX4 (A1933, ABclonal Technology, USA), and *γ*H2AX (ab2893, Abcam, Cambridge, MA, USA). After washing in PBS, the slides were incubated with horseradish peroxidase-labeled secondary antibodies. Five random fields from each slice were observed to count the number of positive cells. Quantitative analysis was performed to obtain the average percentage of positive cells in each field. The results were scored by the same pathologist in a blinded manner.

### 2.5. Periodic Acid Schiff (PAS) Staining

Deparaffinized colon sections were incubated with 1% periodic acid solution (Sigma-Aldrich) and Schiff reagent (Sigma-Aldrich) for 10 min and 40 min, respectively. PAS-stained sections were then counterstained with hematoxylin for 2-5 minutes. The number of PAS-positive cells in each colonic gland was calculated.

### 2.6. Immunofluorescent Staining

The sections of the small intestine and colon were incubated with specific primary anti-IgA antibody (ab223410, Abcam, Cambridge, MA, USA) and anti-ZO-1 antibody (ab96587, Abcam, Cambridge, MA, USA), respectively, overnight at 4°C. Subsequently, the sections were washed 3 times with 1× PBS and incubated with fluorochrome-conjugated secondary antibodies in the dark for 1 h at 37°C. Finally, DAPI (4, 6-diamidino-2-phenylindole, blue, Southern Biotech) was added to the sections to dye the nucleus. Fluorescence photographs were observed using a fluorescence microscope DM5000 B (Leica, Germany).

### 2.7. Real-Time PCR Analysis

Total RNA from intestinal tissues was extracted using the RNeasy mini kit (Qiagen, Carlsbad, CA, USA), and cDNA reverse transcription was performed using the TIANScript RT Kit (Tiangen, Inc., Beijing, China). The endogenous control (glyceraldehyde-3-phosphate dehydrogenase, GAPDH) and oligonucleotide primers for target genes are listed in Table 1. The relative mRNA expression of each target gene including ZO-1, Claudin-1, Occludin, IL-6, IL-1*β*, TNF-*α*, SOD1, SOD2, SIRT1, and PGC1*α* was evaluated using the standard *ΔΔ*Ct method.

### 2.8. Western Blot Analysis

Total proteins of colonic tissues were extracted with RIPA buffer containing protease inhibitors (Solarbio, Beijing, China). The protein concentrations were detected using bicinchoninic acid protein assay (Thermo Scientific Inc.). Proteins were then separated and transferred onto a PVDF membrane (Invitrogen, Carlsbad, CA, USA). The membranes were incubated overnight with the primary antibodies against *β*-actin (ab8226, Abcam, Cambridge, MA, USA), ZO-1 (ab96587, Abcam, Cambridge, MA, USA), CLDN3 (A2946, ABclonal Technology, USA), AMPK (ab32047, Abcam, Cambridge, MA, USA), p-AMPK (Thr172, Cell Signaling Technology), and NF-*κ*B1 (A6667, ABclonal Technology, USA) followed by appropriate secondary antibodies. *β*-Actin was employed as internal controls for total proteins. The intensity of images was determined by ImageJ. Quantitation of band was performed with ImageJ software. All images were converted to 8-bit gray-scale images, and then, a rectangle was drawn around each distinct lane for detection. A profile plot for each band was generated, and then, the intensity of the image was calculated using the area-under-the-curve approach. Three or more replicates were performed and averaged, and statistical significance of differences was obtained by a Student *t*-test.

### 2.9. 16S rRNA Sequencing

Fresh stool samples of 3-week-old and 8-month-old offspring were collected for 16S rRNA gene sequencing. Total fecal bacterial DNA was isolated by QIAamp DNA Stool Mini Kit (QIAamp, Germany), and then, the microbial 16S V3-V4 hypervariable region was amplified. The resulting amplicons were sequenced on an Illumina HiSeq platform (Illumina, San Diego, CA, USA). Optimizing sequences were clustered into operational taxonomic units (OTUs) at ≥97% similarity. Principal component analysis (PCA) was performed on the resulting matrix of distances. R. cluster analysis was carried out to create heatmaps. QIIME platform was used to analyze the alpha/beta diversity. The different species between groups were screened by rank sum test. Based on the Kyoto Encyclopedia of Genes and Genomes (KEGG) database, the microbiota functions were investigated by using Phylogenetic Investigation of Communities by Reconstruction of Unobserved States (PICRUSt). All procedures were performed at TinyGene Bio-Tech (Shanghai) Co., Ltd.

### 2.10. SCFA Quantification

Cecal contents were collected to detect the concentrations of SCFAs (acetate, propionate, butyrate, isobutyrate, valerate, isovalerate, caproate, and heptanoic acid) by gas chromatography (GC) as previously described [23]. Cecal samples were diluted, acidified, and extracted at 0°C for 5 min. Subsequently, the extract was centrifuged at 10 000 rpm and 4°C for 15 min. Liposoluble components in the supernatant were extracted, and the aqueous phase was retained. Then, the aqueous phase was reacted with HCl for 10 min. SCFAs in the aqueous phase were extracted with ethyl acetate. The extract was filtered by 0.22 *μ*m pore-size filter and analyzed by Agilent 7890a series GC. Data were analyzed using Agilent ChemStation software.

### 2.11. Cell Treatment and Gene Silencing of SIRT1

The human intestinal epithelial cell line Caco-2 (ATCC, Manassas, VA, USA) was cultured in Dulbecco's minimum essential media with 20% fetal bovine serum and 1.0% nonessential amino acids. The cells were starved in serum at 37°C for 24 h, then treated with *LGG* supernatant for 24 h.

The small interfering RNA that targets SIRT1 (SIRT1 siRNA; GenePharma, Shanghai, China) was used to knock down the expression of SIRT1. According to the instructions, cells were transfected with 2 *μ*g SIRT1 siRNA or control siRNA. After 6 hours of transfection, the cells were refreshed with medium and then stimulated with the supernatant of live *LGG* or fixed *LGG*.

### 2.12. Data Analysis

SPSS 22.0 (SPSS, Chicago, IL, USA) was used for statistical analysis. The average values were presented as mean ± SEM. One-way ANOVA was applied for multiple comparisons. The two-tailed Student *t*-test was used to define the difference between mean values. *p* < 0.05 was considered a significant statistical difference.

## 3. Results

### 3.1. LGG Colonization in Early Life Promotes Intestinal Development in 3-Week-Old Offspring Mice

The experimental process is shown in Figure 1(a). PCR analysis was performed to detect the colonization of *LGG*, and we found that the specific bands of *LGG* were revealed by the migration spectrum of PCR products from fecal bacterial cultures of 3-week-old mice treated with live *LGG* (Figure 1(b)). The body weight of offspring in the *LGG* colonization group did not differ substantially from that in the control group (Figure 1(c)). The intestinal epithelium is a highly structured tissue composed of repetitive crypt-villus units, and the villi play a critical role in nutrient absorption [24, 25]. We have investigated changes in intestinal architecture and histology to determine the intestinal development of 3-week-old offspring mice. H&E staining showed that treatment with live *LGG* could increase the villus length and crypt depth (Figures 1(d) and 1(e)). Thus, these results indicated that *LGG* colonization in early life promoted the intestinal development of the offspring.

### 3.2. LGG Colonization in Early Life Altered Gut Microbiota Composition in 3-Week-Old Offspring Mice

Next, we used 16S rRNA sequencing to assess the effect of *LGG* colonization in early life on the gut microbiota composition in 3-week-old offspring mice. The Venn diagram was used to show the numbers of shared and unique OTUs between the LC group and the NC group. We found that there were 373 OTUs in the LC group and 345 OTUs in the NC group, with 321 OTUs shared (Figure 2(a)). PCA revealed a clear separation of both groups demonstrating a significant difference in the composition of the gut microbiota (Figure 2(d)). Then, we used the Chao and Shannon diversity index to evaluate the alpha diversity, but we did not see any significant differences in species richness and species diversity between these two groups (Figures 2(b) and 2(c)). To further analyze the discrepancy between groups, beta diversity analysis was performed. The results of nonmetric multidimensional scaling (NMDS) and Jaccard dissimilarity analysis showed that the bacterial community structure segregated differently between the LC group and the NC group (Figures 2(e) and 2(f)). Then, the differentially abundant species at the genus and species level between the LC group and NC group were examined. Interestingly, the relative abundance of *Akkermansia*, *Akkermansia muciniphila*, and SCFA-producing bacteria (*Ruminococcus*, *Coprococcus*, *Odoribacter*, *Faecalibaculum*, and *Lachnospiraceae bacterium A4*) (Figures 2(g) and 2(h)), which have been proved to be positively correlated with longevity, was significantly increased in the LC group.

### 3.3. The Beneficial Effect of LGG Colonization in Early Life on the Microbiota Lasted to 8 Months Old

Venn diagram showed that there were 405 OTUs in the LC group and 419 OTUs in the NC group, with 388 OTUs shared (Figure 3(a)). PCA disclosed that the luminal microbial community in the LC group was significantly different from that in the NC group (Figure 3(b)). Analysis of similarity (ANOSIM) also revealed a significant difference between both groups (*R* = 0.338, *p* = 0.002) (Figure 3(d)). Similar to the results of the gut microbiota analysis of 3-week-old pups, no significant differences were found in the results of alpha diversity between the two groups (Figures 3(e) and 3(f)). When it comes to the beta diversity, PCoA demonstrated that the LC group and NC group were significantly classified into two different groups (Figure 3(c)).

At the phylum level, a previous study showed that the gut microbiota of the elderly was characterized by higher amounts of *Proteobacteria* and decreased amounts of *Firmicutes* and *Actinobacteria* [26, 27]. In our study, the analysis at the phylum level demonstrated that the relative abundance of *Firmicutes* and *Actinobacteria* was elevated in the LC group with the reduction of *Proteobacteria* (Figure 3(g)). The family *Enterobacteriaceae*, which contains a variety of potentially pathogenic microorganisms, was reported to be abundant in the fecal samples of the elderly [4]. Our results showed that the relative abundance of *Enterobacteriaceae* was lower in the LC group than that of the NC group (Figure 3(h)). The microbial composition at the genus and species levels showed that the LC group had higher levels of beneficial bacteria, such as *Lactobacillus*, *Parasutterella*, *Bifidobacterium*, *Akkermansia*, *Akkermansia muciniphila*, and *Lactobacillus intestinalis*, while the opportunistic pathogens such as *Oscillibacter*, *Escherichia*, *Ruminococcus*, *Helicobacter*, and *Alistipes timonensis* showed to be relatively less abundant in the LC group (Figures 4(a)–4(c)).

Furthermore, we determined the changes in the functional composition of the microbiota by using the KEGG pathway database. At KEGG level 1, the proportion of sequences associated with metabolism and genetic information processing was significantly increased in LC group mice (Figure 4(d)). At level 2, the functional categories related to the metabolism of terpenoids and polyketides, replication and repair, and translation were enriched in the fecal microbiome of LC group mice (Figure 4(e)). At level 3, we found that KEGG pathways (including base excision repair, DNA replication, mismatch repair, nucleotide excision repair, tyrosine metabolism, and peptidoglycan biosynthesis) were significantly enriched in LC group mice, and the KEGG pathways (including two-component system, phenylpropanoid biosynthesis, and pentose and glucuronate interconversions) were significantly increased in NC group mice (Figures 4(f) and 4(g)).

### 3.4. LGG Colonization in Early Life Increased the Abundance of SCFA-Producing Bacteria and Production of SCFAs in 8-Month-Old Offspring Mice

The process of aging was accompanied by a decrease in the abundance of SCFA-producing bacteria and the content of SCFAs [28]. Interestingly, at genus and species levels, the abundance of SCFA-producing bacteria in the LC group was higher than that of the NC group, such as *Anaerotruncus*, *Odoribacter*, *Faecalibaculum*, and *Lachnospiraceae bacterium A4* (Figures 4(a)–4(c)). The concentrations of SCFAs (acetate, propionate, butyrate, valerate, isovalerate, and caproate) in cecal contents also significantly increased with the increment of SCFA-producing bacteria in aging mice colonized with live *LGG* (Figure 4(h)). These results showed that *LGG* colonization in early life increased the abundance of SCFA-producing bacteria and the production of SCFAs which might be involved in the protection of aging-related disorders of offspring.

### 3.5. LGG Colonization in Early Life Protected the Intestinal Barrier in 8-Month-Old Offspring Mice

An adequate physical gut barrier consists of a mucous layer, intestinal epithelial cells, and tight junctions [29]. It is pivotal for protection against the potentially harmful compounds and microorganisms while promoting the absorption of nutrients, electrolytes, and water. The process of aging has been confirmed to be accompanied by the destruction of intestinal barrier function [30]. Here, we explored the effect of *LGG* colonization in early life on the intestinal barrier in 8-month-old mice. The goblet cells and tight junction proteins such as ZO-1, Claudin-1, Claudin-3, and Occludin are thought to play critical roles in maintaining gut barrier integrity [23]. IHC staining showed that the number of goblet cells (PAS) and MUC2- (mucin produced by goblet cells) positive cells increased significantly in the experimental group compared with the control group (Figures 5(a) and 5(b)). For the tight junction proteins, our findings indicated that mRNA expression of ZO-1, Claudin-1, and Occludin were upregulated in the LC group (Figure 5(c)). The protein expression levels of ZO-1 and Claudin-3 also showed the same results (Figure 6(a)). Furthermore, immunofluorescence staining showed that *LGG* colonization could increase the membrane localization of ZO-1 (Figure 6(b)).

Immunoglobulin A (IgA) acts as an important first-line barrier that protects the gut epithelium from pathogens and toxins [31]. An increased number of IgA-expressing cells were found in the live-*LGG* group (Figure 6(c)). These data suggested that *LGG* colonization in early life protected the intestinal barrier in the early phase of aging mice.

### 3.6. LGG Colonization in Early Life Enhanced Age-Related Antioxidant Defense and Weakened DNA Damage in 8-Month-Old Offspring Mice

Increased resistance to oxidative stress has been shown to improve longevity. Superoxide dismutase (SOD) is an important component of the antioxidant defense system [32]. The mRNA expression level of SOD1 and SOD2 in colon tissues was dramatically higher in the LC group mice relative to the NC group mice (Figure 7(a)).

Glutathione peroxidase (GPX) family is a major member of the antioxidant enzyme family, and its activity decreases with age [33]. We evaluated the expression of GPX4 in the colon tissues in 8-month-old offspring by immunohistochemistry. We found that the expression of GPX4 in the *LGG* colonization group significantly increased than that in the control group (Figure 7(b)). Oxidative stress can cause DNA damage which is closely related to aging [34, 35]. The *γ*-H2AX immunohistochemistry revealed significantly decreased DNA damage in the colon epithelial cells of aging mice colonized with live *LGG* compared to noncolonized (Figure 7(c)).

### 3.7. LGG Colonization in Early Life Inhibited Intestinal Low-Grade Inflammation in 8-Month-Old Offspring Mice

The chronic low-grade inflammation during aging is closely related to age-related diseases [36]. No obvious microscope inflammation in two groups was observed. The relative mRNA expression levels of proinflammatory factors (IL-1*β*, IL-6, and TNF-*α*) were significantly decreased in the LC group relative to the NC group (Figure 7(a)). Therefore, *LGG* colonization in early life might attenuate inflammaging of offspring.

### 3.8. LGG Colonization in Early Life Activated the SIRT1/AMPK/PGC-1*α* Pathway

SIRT1, an NAD^+^-dependent deacetylase, has been identified as an antiaging molecule [37]. AMPK and SIRT1 are present in all eukaryotic cells and are closely linked in regulating inflammation. Activation of SIRT1 leads to phosphorylation of AMPK [38]. PGC-1*α*, which acts as an important downstream target of the SIRT1/AMPK pathway, has shown anti-inflammatory potential by inhibiting the activity of NF-*κ*B [39]. In our study, the mRNA levels of SIRT1 and PGC-1*α* and protein expression level of p-AMPK increased significantly in the LC group compared with that in the NC group, while the expression of NF-*κ*B showed a downward trend (Figures 8(a)–8(c)).

### 3.9. The Protective Effect of LGG Was Blunted after SIRT1 Gene Silencing in Intestinal Epithelial Cells

Compared with the control group, the mRNA expression levels of SIRT1 and PGC-1*α* in Caco2 cells treated with *LGG* supernatant were significantly increased (Figures 8(d) and 8(e)). Furthermore, we explored the vital role of SIRT1 through siRNA-mediated silencing of the gene encoding SIRT1. The results showed that the silencing of SIRT1 blocked the *LGG*-mediated upregulation of SIRT1 and PGC-1*α* in Caco2 cells (Figures 8(d) and 8(e)). Collectively, these data indicated that *LGG*-induced activation of the SIRT1/AMPK/PGC-1*α* pathway may be a critical mechanism for antiaging effects.

## 4. Discussion

Aging is defined as a biological process in which physiological functions are gradually impaired. Recently, studies have documented the crucial role of the microbial community in the host aging process [40–42]. Supplementation of probiotics in elderly populations, particularly those containing *Lactobacillus* or *Bifidobacterium*, appears to be a promising intervention to delay senescence [43–45]. The gut microbiota in early life participates in a range of biological processes of the host including immunity, cognitive neurodevelopment, and metabolism [46]. The intervention of probiotics in the aging stage has shown beneficial effects on the host, but their colonization in early life may be a more effective and long-lasting solution. As demonstrated in our study, *LGG* colonization in early life could protect the intestinal barrier, modulate gut microbiota dysbiosis, enhance antioxidant defense, weaken DNA damage, and inhibit low-grade inflammation in the early phase of aging of offspring. In addition, the mechanisms involved in the protective effects might be related to the activation of the SIRT1/AMPK/PGC-1*α* pathway and repression of NF-*κ*B (Figure 9). Therefore, *LGG* colonization in early life might play a protective role during the aging process of offspring.

Normal intestinal villus is an important part of barrier function, which is essential for digestion and absorption [4]. It is commonly accepted that decreased villus height/width and density can be found in the small intestine tissues of aging rats [47–49]. In our study, we found that *LGG* colonization in early life positively impacts the intestinal development of offspring. In recent years, there has been an increasing amount of evidence showing that the integrity of the intestinal epithelial barrier function was critical for maintaining health and homeostasis [50]. Disruption of the intestinal barrier is involved in intestinal and extraintestinal diseases [51]. The aging process was accompanied with the malfunctioning of the intestinal barrier [30], which was closely associated with activation of inflammatory pathways and age-related disorders, such as Parkinson's disease and Alzheimer's disease [52–55]. Tight junctions between epithelial cells act as a key factor contributing to the maintenance of normal barrier function. The molecular compositions of the tight junctions mainly consist of ZO-1, Occludin, Claudin, and junctional adhesion molecules [49]. As reported by Tran and Greenwood-Van [30], decreased expression of ZO-1 and Occludin in colonic tissues from old baboons was observed. Our results showed that *LGG* colonization in early life has beneficial effects on the intestinal barrier function and integrity in the early phase of aging mice.

Recently, a considerable literature has grown up around the theme of gut microbiota during aging. The effects of aging on alpha diversity remain obscure. Initially, it was found that alpha diversity decreased during aging [56, 57]. However, several studies have shown that the microbial population of the elderly has a higher alpha diversity [58–60], or no significant difference [26, 61], compared with the younger adults. This may be due to various confounding factors affecting the alpha diversity of the microbiome, including host or lifestyle factors [4]. Data from our study showed no significant difference in alpha diversity between the LC group and NC group. The abnormal changes in the gut microbiota diversity were closely related to aging-related disorders [62]. Probiotic supplementation has shown great potential in counteracting age-related shifts in gut microbiota composition and diversity and then impacting health outcomes and promoting healthy aging [11]. Many studies have confirmed a decrease abundance of *Bifidobacteria* in the fecal samples of the elderly [63–65]. However, it has been reported that the abundance of *Bifidobacteria* may fluctuate with the increasing age. The abundance of *Bifidobacteria* in feces of centenarians (99-104 years old) decreased compared with that of young adults or elderly (>65 years old) but increased in (super) centenarians (>105 years old) [4]. *Bifidobacteria* has been shown to participate in innate and adaptive immune processes to maintain immune homeostasis [66]. Along this line, our data demonstrated that *LGG* colonization in early life can increase the abundance of beneficial bacteria, especially *Bifidobacteria*, which may contribute to its inhibitory impact on aging by regulating immunity.

*Akkermansia muciniphila* is a mucin-degrading bacteria that is highly enriched in the colon of healthy individuals. It can competitively inhibit the degradation of mucin by other pathogens [67, 68]. *Akkermansia muciniphila* has shown great potential in improving host metabolic function and immune response [69]. *Akkermansia muciniphila*-like bacteria was colonized in the intestine in early life and developed to a level close to that of adults within one year but decreased significantly in the elderly [70]. However, both clinical and animal studies have confirmed that the abundance of *Akkermansia muciniphila* decreased or even disappeared completely during aging [22, 26, 71, 72]. Interestingly, semisupercentenarians (105-109 years old) were characterized by an increasing abundance of *Akkermansia* spp than younger elderly people [65]. It is known that *Akkermansia muciniphila* has important value in improving host metabolic function and immune response [69]. Data from our study showed that *LGG* colonization in early life could increase the abundance of *Akkermansia muciniphila* in 8-month-old offspring mice. However, more in-depth work is needed to explore the underlying mechanisms of the microbial modulation.

SCFAs, the main metabolites generated by gut bacterial fermentation of dietary fibre, were negatively correlated with inflammatory conditions, specifically in senescence [73]. A variety of bacteria including *Akkermansia muciniphila* promoted the production of SCFAs [67, 74]. The reduction of SCFAs in the intestine is one of the important manifestations related to aging [75–77]. In addition, SCFAs could provide energy for colon epithelial cells, maintain intestinal barrier function, and regulate immune response [78, 79]. Butyrate, the most common study object of SCFAs in intestinal health, has been found to extend the lifespan by inhibiting the histone deacetylase activity [80]. In this study, we observed that *LGG* colonization in early life increased the abundance of SCFA-producing bacteria, together with the production of SCFAs in the early phase of aging mice. These findings suggested that *LGG* colonization in early life may promote the production of SCFAs.

The sirtuins are highly conserved NAD^+^-dependent protein deacetylases/ADP ribosyltransferases, including Sir2 found in yeast cells and its homologous analogues SIRT1 to SIRT7 in mammals [81, 82]. SIRT1 is the most comprehensively studied protein molecule related to aging in the sirtuin family. Activation of SIRT1 was thought to be protective against age-related diseases, including the ability to improve glucose tolerance, inhibit tumor progression, and regulate the metabolism of lipid and cholesterol [83]. Over the past few years, SIRT1 has been proven to play a critical role in the suppression of inflammation [82, 84]. In addition, the increased expression of NF-*κ*B during aging can induce oxidative stress and inflammation [85, 86]. SIRT1 can suppress inflammation by inhibiting NF-*κ*B partly through activating AMPK and PGC-1*α* [39]. Interestingly, we found that *LGG* could activate the SIRT1/AMPK/PGC-1*α* pathway and repressed the expression of NF-*κ*B. Therefore, we speculate that the activation of the SIRT1/AMPK/PGC-1*α* signaling pathway plays a key role in *LGG* ameliorating inflammaging.

Taken together, this study offers an insight into the understanding of how *LGG* colonization in early life can ameliorate inflammaging of offspring, including protecting the intestinal barrier, increasing the abundance of beneficial bacteria, promoting the production of SCFAs, and activating the SIRT1/AMPK/PGC-1*α* signaling pathway. This would provide a new strategy for the prevention of age-related diseases.

## 5. Conclusions

*LGG* colonization in early life could rebalance the gut microbiota, increase the production of cecal SCFAs, protect intestinal barrier, enhance antioxidant defense, attenuate epithelial cell DNA damage, inhibit intestinal low-grade inflammation, and activate the SIRT1/AMPK/PGC-1*α* pathway in the early phase of aging mice. Thus, *LGG* colonization in early life may have beneficial effects on delaying aging-related disorders.

## Figures and Tables

**Figure 1:** *Lactobacillus rhamnosus GG* colonization in early life protected intestinal development of 3-week-old offspring. (a) The experimental process of this study. (b) DGGE technology was used to identify the colonization of *LGG* in 3-week-old offspring. (c) The changes in body weight throughout the experiment. (d, e) HE staining was performed to detect the villus length or crypt depth of the intestine in 3-week-old offspring. *LGG*: *Lactobacillus rhamnosus GG*; DGGE: denaturing gradient gel electrophoresis; LC: *LGG* colonization, *n* = 7; NC: noncolonization, *n* = 7. Scale bar: 50 *μ*m. ^∗∗^*p* < 0.05, ^∗∗^*p* < 0.01, and ^∗∗∗^*p* < 0.001.

**Figure 2:** *Lactobacillus rhamnosus GG* colonization in early life altered specific bacterial taxa in 3-week-old offspring mice. (a) Venn diagram showed the intersection of the bacterial OTUs. (b, c) The alpha (Chao and Shannon index) diversity was shown. (d) Results from PCA are shown. (e, f) To compare the beta diversity among the groups, NMDS and Jaccard dissimilarity analysis were performed. (g, h) Key bacterial changes at the phylum, class, order, family, and genus levels. PCA: principal component analysis; NMDS: nonmetric multidimensional scaling. *LGG* colonization, *n* = 6. Noncolonization, *n* = 6.

**Figure 3:** *Lactobacillus rhamnosus GG* colonization in early life altered the composition and diversity of gut microbiota in 8-month-old offspring mice. (a) The Venn diagram was drawn to describe the overlapping OTUs between the two groups. (b, c) PCA and PCoA of the bacterial population structures. (d) Analysis of similarity (ANOSIM) test. (e, f) Alpha diversity was calculated using the ace and Shannon index. (g, h) Gut microbiota analysis at phylum and family levels. PCA: principal component analysis; PCoA: principal coordinate analysis; *LGG* colonization, *n* = 7. Noncolonization, *n* = 7.

**Figure 4:** *Lactobacillus rhamnosus GG* colonization in early life increased the abundance of beneficial bacteria and promoted short-chain fatty acid production in 8-month-old offspring mice. (a, b) Gut microbiota analysis at genus and species levels. (c) Linear discriminant analysis effect size (LEfSe) analysis was performed to identify differentially enriched bacteria. (d–g) Plots of KEGG pathway comparisons between the *LGG*-colonization group and noncolonization group at level 1, level 2, and level 3. (h) Detection of concentrations of SCFAs (acetate, propionate, butyrate, isobutyrate, and valerate) in cecal contents. SCFAs: short-chain fatty acids; LC: *LGG* colonization, *n* = 7; NC: noncolonization, *n* = 7.

**Figure 5:** *Lactobacillus rhamnosus GG* colonization in early life protected the intestinal barrier in 8-month-old offspring mice. (a) Periodic acid Schiff staining was performed to detect the goblet cells in the colon. (b) Immunohistochemical detection of MUC2 in colon tissues. The number of positive cells was assessed. (c) The relative mRNA level of ZO-1, Claudin-1, and Occludin was detected by real-time PCR. *LGG*: *Lactobacillus rhamnosus GG*. *LGG* colonization, *n* = 7. Noncolonization, *n* = 7. Scale bar: 50 *μ*m. ^∗∗^*p* < 0.05, ^∗∗^*p* < 0.01, and ^∗∗∗^*p* < 0.001.

**Figure 6:** *Lactobacillus rhamnosus GG* colonization in early life protected tight junction in the colon and increased IgA in the small intestine in 8-month-old offspring mice. (a) Western blot analysis was performed to assess the protein expression of ZO-1 and CLDN3. (b, c) Detection of ZO-1 in colonic tissues and IgA in the small intestine by immunofluorescent staining. *LGG*: *Lactobacillus rhamnosus GG*. *LGG* colonization, *n* = 7. Noncolonization, *n* = 7. Scale bar: 50 *μ*m. ^∗^*p* < 0.05 and ^∗∗∗^*p* < 0.001.

**Figure 7:** *Lactobacillus rhamnosus GG* colonization in early life improved the antioxidant defense and inhibited low-grade intestinal inflammation in 8-month-old offspring mice. (a, b) Real-time PCR analysis and immunohistochemical detection of inflammatory factors (IL-1*β*, IL-6, and TNF-*α*) and antioxidant markers (SOD1, SOD2, and GPX4). (c) The *γ*-H2AX staining in colon tissues to assess the DNA damage. *LGG* colonization, *n* = 7. Noncolonization, *n* = 7. Scale bar: 50 *μ*m. ^∗^*p* < 0.05, ^∗∗^*p* < 0.01, and ^∗∗∗^*p* < 0.001.

**Figure 8:** *Lactobacillus rhamnosus GG* colonization in early life activated the SIRT1/AMPK/PGC-1*α* pathway and decreased NF-*κ*B expression. (a, b) Relative mRNA expression of SIRT1 and PGC-1*α* in colon tissues. (c) The protein levels of total and phosphorylated AMPK and NF-*κ*B were detected by western blotting, and the relative intensity was quantified by ImageJ software. (d, e) Expression of SIRT1 and PGC-1*α* in SIRT1-knockdown Caco2 cells relative to the negative control. *LGG* colonization, *n* = 7. Noncolonization, *n* = 7. ^∗^*p* < 0.05, ^∗∗^*p* < 0.01, and ^∗∗∗^*p* < 0.001.

**Figure 9:** *Lactobacillus rhamnosus GG* colonization in early life ameliorates inflammaging of offspring. *LGG* colonization in early life significantly protected intestinal barrier function, enhanced antioxidant defense, and attenuated epithelial cell DNA damage in the early phase of aging mice. Decreased proinflammatory factors indicated that low-grade inflammatory was inhibited in the *LGG* colonization group. Interestingly, fecal microbiota analysis showed that the composition and diversity were significantly different between the two groups. Longevity-related bacteria (*Akkermansia muciniphila*, *Lactobacillus*, and *Bifidobacterium*) increased significantly in the *LGG* colonization group. *LGG* colonization increased the abundance of SCFA-producing bacteria and the content of cecal SCFAs. In addition, *LGG* plays an anti-inflammaging effect by activating the SIRT1/AMPK/PGC-1*α* pathway. TJ: tight junctions; IgA: immunoglobulin A; IL-1*β*: interleukin 1*β*; IL-6: interleukin 6; TNF-*α*: tumor necrosis factor-*α*; SCFAs: short-chain fatty acids.

**Table 1:** Primer sequences used for real-time PCR.

Primers	Sequence
GAPDH	Forward 5′-GGAGAAACCTGCCAAGTATG-3′
	Reverse 5′-TGGGAGTTGCTGTTGAAGTC-3′
ZO-1	Forward 5′-GGGCCATCTCAACTCCTGTA-3′
	Reverse 5′-AGAAGGGCTGACGGGTAAAT-3′
Claudin-1	Forward 5′-AGACCTGGATTTGCATCTTGGTG-3′
	Reverse 5′-TGCAACATAGGCAGGACAAGAGTTA-3′
Occludin	Forward 5′-CGGTACAGCAGCAATGGTAA-3′
	Reverse 5′-CTCCCCACCTGTCGTGTAGT-3′
IL-1*β*	Forward 5′-GTGGCTGTGGAGAAGCTGTG-3′
	Reverse 5′-GAAGGTCCACGGGAAAGACAC-3′
IL-6	Forward 5′-CCAGTTGCCTTCTTGGGACT-3′
	Reverse 5′-GGTCTGTTGGGAGTGGTATCC-3′
TNF-*α*	Forward 5′-ACTCCAGGCGGTGCCTATG-3′
	Reverse 5′-GAGCGTGGTGGCCCCT-3′
SOD1	Forward 5′-TGTGTCCATTGAAGATCGTGTG-3′
	Reverse 5′-TCCCAGCATTTCCAGTCTTTG-3′
SOD2	Forward 5′-TGCTCTAATCAGGACCCATTG-3′
	Reverse 5′-CATTCTCCCAGTTGATTACATTCC-3′
SIRT1	Forward 5′-CTCTGAAAGTGAGACCAGTAGC-3′
	Reverse 5′-TGTAGATGAGGCAAAGGTTCC-3′
PGC-1*α*	Forward 5′-TATGGAGTGACATAGAGTGTGCT-3′
	Reverse 5′-CCACTTCAATCCACCCAGAAAG-3′

## Data Availability

The data that support the findings of this study are openly available in Sequence Read Archive (SRA) of NCBI at http://www.ncbi.nlm.nih.gov/bioproject/743142, reference number PRJNA743142.
